The article "Discriminative Codebook Hashing for Supervised Video Retrieval" was published in 2021. Journal: Comput Intell Neurosci.

# Discriminative Codebook Hashing for Supervised Video Retrieval

**DOI:** 10.1155/2021/5845094

**Published:** 2021-08-25

**Authors:** Xiaoman Bian, Rushi Lan, Xiaoqin Wang, Chen Chen, Zhenbing Liu, Xiaonan Luo, Kuei-Kuei Lai

**Affiliations:** ^1^Guangxi Key Laboratory of Image and Graphic Intelligent Processing, Guilin University of Electronic Technology, Guilin 541004, China; ^2^Department of Business Administration, Chaoyang University of Technology, Taichung 413310, Taiwan, China

## Abstract

In recent years, hashing learning has received increasing attention in supervised video retrieval. However, most existing supervised video hashing approaches design hash functions based on pairwise similarity or triple relationships and focus on local information, which results in low retrieval accuracy. In this work, we propose a novel supervised framework called discriminative codebook hashing (DCH) for large-scale video retrieval. The proposed DCH encourages samples within the same category to converge to the same code word and maximizes the mutual distances among different categories. Specifically, we first propose the discriminative codebook via a predefined distance among intercode words and Bernoulli distributions to handle each hash bit. Then, we use the composite Kullback–Leibler (KL) divergence to align the neighborhood structures between the high-dimensional space and the Hamming space. The proposed DCH is optimized via the gradient descent algorithm. Experimental results on three widely used video datasets verify that our proposed DCH performs better than several state-of-the-art methods.

## 1. Introduction

Under the condition of the increase in smartphones, the amount of video data has shown an explosive growth trend [1–3]. For example, TikTok has over 400 million daily active users who upload approximately 2,000 videos every minute. YouTube receives a total of 100 hours of videos per minute [4–6]. Due to the economic storage and efficiency of binary codes, hash-based methods have been widely applied to visual retrieval tasks [7–13].

Previous hash-related work [14] mainly focused on image hashing and can be divided into data-independent and data-dependent methods. Data-independent approaches learn binary codes without data information but through random space projection. The most representative algorithm is local sensitive hashing (LSH) [15], which generates huge redundant information using random mapping and obtains satisfactory performance with long hash codes. Data-dependent hash methods [16–18], which can also be divided into unsupervised hashing and supervised hashing, are proposed to generate more efficient hash codes by maintaining the neighborhood structure between data. For example, Gong et al. [19] proposed iterative quantization hashing (ITQ), which minimizes quantization error by rotating principal component analysis (PCA) projection data. Spectral hashing (SH) [20] assumes that data obey a uniform distribution and divides the data according to the main direction of the data stream. Density sensitive hashing (DSH) [21] extends LSH by studying structural information. Zhang et al. [22] developed a convergence-preserving parametric learning algorithm, called latent factor hashing (LFH), to learn similarity-preserving binary codes based on latent factor models. Liu et al. [23] proposed kernel supervised hashing (KSH) by applying kernel-based formulas to accommodate linearly inseparable data and designed a greedy algorithm to solve the hash function optimization problem.

In recent years, hashing methods proposed for video retrieval have also received extensive attention [24–31] and are composed of two categories: machine learning methods and deep hashing. Machine learning methods, resembling image hashing approaches, learn binary codes of video keyframes based on the low-level manual features and then calculate video hashing codes via averaging. Wu et al. [4] employed video hashing via using color histograms to obtain global features. This is the first application of hash learning in the video field. Multiple-feature hashing (MFH) [32] adopts the weight-based method to combine different features. Ye et al. [33] used video structural information in the supervised learning paradigm to obtain the optimal binary codes. Stochastic multiview hashing (SMVH) [34] attempts to separately calculate the probability similarity matrices of video frames in the feature space and the Hamming space, and then, the difference between the above two probability matrices is minimized using the KL divergence. Nie et al. [35] defined joint multiview hashing (JMVH) by maximizing the interclass distance and minimizing the innerclass distance to preserve the global structure and local structure with multiple features. Boosting temporal video hashing (BTVH) [36] studies the multitable learning problem to boost the performance and captures the inherent similarity of video from both visual and temporal perspectives. In addition, some researchers in recent years have used deep networks to obtain the temporal and spatial information between keyframes. For instance, central similarity quantization (CSQ) [37] learns the temporal information by using 3D convolutional neural networks and proposes a view point called hash center to enhance the central similarity.

However, most existing video hashing approaches may lead to the following problems. (1) Low discriminability among different categories: functions based on pairwise similarity or triple relationships only consider local information, which results in good maintenance of the information of similar samples but shows poor performance in distinguishing samples from different categories. (2) Poor performance in real-world scenarios: in real application scenarios, similar data often accounts for only a small proportion, and most samples are not similar, which leads to low efficiency when the data are imbalanced [37]. (3) Greater time costs on deep learning: deep learning frameworks are time-consuming when training models and have no significant performance based on the spatiotemporal information extracted by the network. Hence, these video hashing functions cannot learn discriminative hash codes to enhance the performance.

To solve the above problems, in this work, we propose a novel framework for supervised video retrieval, called discriminative codebook hashing, which considers the global structure to construct the hash function. DCH encourages samples within the same category to converge to the identical codeword and maximizes the mutual distances between different categories. Specifically, the discriminative codebook is first generated based on two characters: the predefined distance between intercode words and Bernoulli distributions for ensuring that each hash bit stores more information. Then, to keep the similarity matrix between the feature space and the Hamming space, the composite KL divergence is proposed to solve this problem. Finally, the gradient descent algorithm is utilized to optimize the algorithm. In this way, we can obtain discriminative binary codes for video retrieval.  Figure 1 shows the framework of DCH, and the method we proposed has the following innovations:

- We proposed the discriminative codebook based on the predefined distance between intercode words and Bernoulli distributions for ensuring each hash bit to store more information
- The DCH method, which can maximize the distance of the intercode words generated by the predefined codebook to learn discriminative binary codes for supervised video retrieval, is proposed
- We verify our proposed method by experimenting on three widely used datasets, which shows that DCH has a significant improvement in contrast with several state-of-the-art methods

The other sections are organized as follows.  Section 2 introduces some preliminary works.  Section 3 introduces the proposed discriminative codebook hashing in detail. The experimental work is presented in Section 4, and the conclusion of DCH is shown in Section 5.

## 2. Preliminary Work

In this section, we briefly introduce the preliminary work, namely, stochastic multiview hashing [34]. It is a supervised video retrieval method that aims to preserve the similarity structure from the original space to the Hamming space.

Let *V*={*v*_*i*_}_*i*=1_^*n*_*v*_^ be the video set, where *v*_*i*_ indicates the *i*th video of *V* and *n*_*v*_ is the number of videos. *H*={*h*_*i*_}_*i*=1_^*n*_*v*_^ is hash code of the video set, where *h*_*i*_ ∈ {0,1} is *l*-bit length binary codes transformed by *v*_*i*_. The video features are extracted based on the set of keyframe features *X*={*x*_*i*_}_*i*=1_^*n*^, where *x*_*i*_ ∈ ℝ^1×*d*^, *n* is the number of keyframes, and *d* is the dimension of each keyframe. *Z*={*z*_*i*_}_*i*=1_^*n*^ represents the corresponding binary codes of the keyframes, where *z*_*i*_ ∈ ℝ^1×*l*^. The conversion relationships between the above variables are formulated as

(1) $$\begin{array}{c} \tilde{Z}=XW+b, \end{array}$$

(2) $$\begin{array}{c} Z=\text{sigmoid}\left(\tilde{Z}\right), \end{array}$$

(3) $$\begin{array}{c} h_{i}=T\left(\frac{1}{\left|{\text{Ind}}_{i}\right|}\sum_{j\in {\text{Ind}}_{i}}z_{j\cdot }\right), \end{array}$$

where $\tilde{Z}\in {\mathbb{R}}^{n\times l}$ is the temporal result of linear projection, *b* ∈ ℝ^*l*^ is a bias parameter, *W* ∈ ℝ^*d*×*l*^ is the projection matrix, Ind_*i*_ is the set of frames, and |Ind_*i*_| is the sum of samples in the set. The high-dimensional keyframe feature matrix *X* is first projected into the lower matrix $\tilde{Z}$. Then, the sigmoid function is used to map the variable between 0 and 1. Finally, a thresholding function is used to change the data into a binary code with *T*(*y*)=0 if *y* < 0.5 and *T*(*y*)=1, otherwise.

SMVH keeps the similarity matrix between the feature space and the Hamming space using a composite KL divergence measure. In particular, it separately calculated the similarity probability matrix *P* in the original space and the pairwise similarity matrix *Q* among samples in the Hamming space. Then, the KL divergence is used to examine how well the above two probability matrices *P* and *Q* match. Therefore, the objective function of SMVH is defined as follows:

(4) $$\begin{array}{c} \underset{W,b}{\min}\;S_{\text{KL}}\left(W,b\right)+\frac{\mu }{2}{\left\|W\right\|}_{F}^{2}, \end{array}$$

where *μ* > 0 controls the weight of the regular term to prevent overfitting and *S*_KL_(*W*, *b*) is the composite KL divergence. The latter can be represented as

(5) $$\begin{array}{c} S_{\text{KL}}\left(W,b\right)=\lambda \text{KL}\left(\left.P\;\right\|\;Q\right)+\left(1-\lambda \right)\text{KL}\left(\left.Q\;\right\|\;P\right), \end{array}$$

where 0  ≤  *λ*  ≤ 1 controls the influence of the composite KL divergence, *P*={*p*_*i*_}_*i*=1_^*n*^ ∈ ℝ^*n*×*n*^ is the similarity structure based on *X*, and *Q*={*q*_*i*_}_*i*=1_^*n*^ ∈ ℝ^*n*×*n*^ is another probability matrix preserving the similarity information of *Z* in the Hamming space. In addition, the KL divergence is defined as follows:

(6) $$\begin{array}{c} \text{KL}\left(\left.P\;\right\|\;Q\right)=\sum_{i=1}^{n}\sum_{j\neq i}p_{j|i}\log\frac{p_{j|i}}{q_{j|i}}, \end{array}$$

where *p*_*j|i*_ is a conditional probability that reflects the similarity between *x*_*i*_ and *x*_*j*_, and another conditional probability *q*_*j|i*_ represents the probability of returning *z*_*j*_ given the query *z*_*i*_.

## 3. Discriminative Codebook Hashing

In this section, we present the proposed DCH in detail through four parts, including the proposed discriminative codebook, the objective function, algorithmic optimization, and complexity analysis.

### 3.1. Discriminative Codebook

Motivated by CSQ [37], we propose a novel and discriminative codebook *C*={*c*_*i*_}_*i*=1_^*m*^ for supervised video retrieval, where *c*_*i*_ ∈ {0,1}^1×*l*^ is the code word of the *i*th category. The proposed codebook is defined according to two characters. The first is that the value in the same bit of different code words obeys a Bernoulli distribution. Specifically, the proportions of 0 and 1 of the same bit in different categories are both 50%, that is, *c*_·*i*_ has a 50% probability of being 0 or 1, which will maximize the entropy and store more information in each bit. The other is that the mutual distances among intercode words are defined as follows:

(7) $$\begin{array}{c} D_{H}\left(c_{i},c_{j}\right)\geq \frac{l}{2}-f, \end{array}$$

where *D*_*H*_ is the Hamming distance between code words *c*_*i*_ and *c*_*j*_, *l* is the length of binary codes, and *f* represents the fault tolerance. The mutual distance between intercode words will be the largest constrained by equation (7).

Overall, the proposed codebook encourages samples within the same category to converge to the same codeword and maximizes the mutual distance between different categories. Therefore, the proposed codebook can preserve global structures and help generate discriminative binary codes for video retrieval. The scheme of the proposed discriminative codebook is presented in Algorithm 1.

### 3.2. Objective Function

According to the proposed discriminative codebook *C*, we expand each row of the codebook matrix *C* into *R*={*r*_*i*_}_*i*=1_^*n*^ according to the number of samples, where *r*_*i*_ ∈ ℝ^1×*l*^. The detailed generation process of *R* is shown in Algorithm 2. We minimize the error between the binary codes and the predefined codebook as

(8) $$\begin{array}{c} \underset{W,b}{\min}{\left\|Z-R\right\|}_{F}^{2}. \end{array}$$

Specifically, for each *z*_*i*_ ∈ *Z*, we take *r*_*i*_ as the codebook of *z*_*i*_ ∈ *Z* to make samples in the same category share the same codebook and samples in different categories have discriminative binary codes.

To keep the similarity matrix between the feature space and the Hamming space, we join the composite KL divergence and our proposed codebook to construct the overall objective function of DCH as follows:

(9) $$\begin{array}{c} \underset{W,b}{\min}\;S_{\text{KL}}\left(W,b\right)+\frac{\gamma }{2}{\left\|Z-R\right\|}_{F}^{2}+\frac{\mu }{2}{\left\|W\right\|}_{F}^{2}, \end{array}$$

where *γ* controls the weight of the error loss between the codebook and the learned hash codes, and the second term of equation (9) aligns values between binary codes and their corresponding code word.

In this way, our proposed DCH can solve the problem that other algorithms only consider the pairwise relationships and ensure that samples in the same category share the same code word. Furthermore, DCH maximizes the mutual distances between different categories and then obtains discriminative binary codes.

### 3.3. Algorithmic Optimization

The optimization problem has two main variables: *W* and *b*. Our solution is to use the gradient descent algorithm to find good solutions. To facilitate the writing, we split the objective function equation (9) into three parts:

(10) $$\begin{array}{c} \Phi_{1}\left(W,b\right)=S_{KL}\left(W,b\right),\\ \Phi_{2}\left(W,b\right)=\frac{\gamma }{2}{\left\|Z-R\right\|}_{F}^{2},\\ \Phi_{3}\left(W\right)=\frac{\mu }{2}{\left\|W\right\|}_{F}^{2}. \end{array}$$

The detailed optimization procedure is presented as follows.

**W-Step**: the corresponding problem is to minimize the following loss function:

(11) $$\begin{array}{c} \underset{W}{\min}\;S_{\text{KL}}\left(W,b\right)+\frac{\gamma }{2}{\left\|Z-R\right\|}_{F}^{2}+\frac{\mu }{2}{\left\|W\right\|}_{F}^{2}. \end{array}$$

To compute the optimal *W*, the relevant deviation formula can be expressed as

(12) $$\begin{array}{c} \text{d}W=\frac{\partial \Phi_{1}\left(W,b\right)}{\partial W}+\frac{\partial \Phi_{2}\left(W,b\right)}{\partial W}+\frac{\partial \Phi_{3}\left(W\right)}{\partial W}. \end{array}$$

The derivative of ∂Φ_1_(*W*, *b*) w.r.t. *W* can be computed as follows:

(13) $$\begin{array}{c} \frac{\partial \Phi_{1}\left(W,b\right)}{\partial W}={\left[\frac{\partial \Phi_{1}\left(W,b\right)}{\partial z_{ik}}\frac{\partial z_{ik}}{\partial w_{kj}}\right]}_{d\times l}, \end{array}$$

where ∂Φ_1_(*W*, *b*)/∂*z*_*ik*_ and ∂*z*_*ik*_/∂*w*_*kj*_ are represented as

(14) $$\begin{array}{c} \frac{\partial \Phi_{1}\left(W,b\right)}{\partial z_{ik}}=2\left(\lambda \left(p_{i|t}-q_{i|t}+p_{t|i}-q_{t|i}\right)+\left(1-\lambda \right)*\right.\left(q_{t|i}\sum_{g\neq i}q_{g|i}\log\frac{q_{g|i}}{p_{g|i}}+q_{i|t}\sum_{g\neq t}q_{g|t}\log\frac{q_{g|t}}{p_{g|t}}-\log\frac{q_{t|i}}{p_{t|i}}-\log\frac{q_{i|t}}{p_{i|t}}\right)\left(z_{ik}-z_{tk}\right),\\ \frac{\partial z_{ik}}{\partial w_{kj}}=z_{ik}\left(1-z_{ik}\right)x_{ji}. \end{array}$$

Following the norm derivation law, ∂Φ_2_(*W*, *b*)/∂*W* can be optimized as follows:

(15) $$\begin{array}{c} \frac{\partial \Phi_{2}\left(W,b\right)}{\partial W}=\frac{\partial \Phi_{2}\left(W,b\right)}{\partial Z}\frac{\partial Z}{\partial W}=X^{T}\left(\left(Z-R\right)⊙\left(Z⊙\left(1-Z\right)\right)\right), \end{array}$$

where ⊙ indicates that the elements in the same position of two matrices are multiplied.

For ∂Φ_3_(*W*)/∂*W*, we have the derivative that

(16) $$\begin{array}{c} \frac{\partial \Phi_{3}\left(W\right)}{\partial W}=\mu W. \end{array}$$

**b-Step**: the subproblem of *b* is given by

(17) $$\begin{array}{c} \underset{b}{\min\;}S_{KL}\left(W,b\right)+\frac{\gamma }{2}{\left\|Z-R\right\|}_{F}^{2}. \end{array}$$

The deviation w.r.t. *b* can be expressed as

(18) $$\begin{array}{c} \text{d}b=\frac{\partial \Phi_{1}\left(W,b\right)}{\partial b}+\frac{\partial \Phi_{2}\left(W,b\right)}{\partial b}. \end{array}$$

The derivative of ∂Φ_1_(*W*, *b*)/∂*b* is described as follows:

(19) $$\begin{array}{c} \frac{\partial \Phi_{1}\left(W,b\right)}{\partial b}={\left[\frac{\partial \Phi_{1}\left(W,b\right)}{\partial z_{ik}}\frac{\partial z_{ik}}{\partial b_{k}}\right]}_{1\times l}, \end{array}$$

where

(20) $$\begin{array}{c} \frac{\partial z_{ik}}{\partial b_{k}}=z_{ik}\left(1-z_{ik}\right). \end{array}$$

The second term of equation (18) is described as follows:

(21) $$\begin{array}{c} \frac{\partial \Phi_{2}\left(W,b\right)}{\partial b}=\frac{\partial \Phi_{2}\left(W,b\right)}{\partial Z}\frac{\partial Z}{\partial b}=\left(Z-R\right)⊙\left(Z⊙\left(1-Z\right)\right). \end{array}$$

Algorithm 2 describes the overall algorithm optimization process of the proposed DCH.

### 3.4. Complexity Analysis

The time complexity of the entire training process of SMVH [34] is approximately *O*(*Tn*^3^+*n*^2^), and the proposed DCH algorithm adds two parts time-consuming on this basis. The first part is the learning process of *C*, and the time complexity is *O*(*T*_*c*_*l*). The second part is that the time complexity of optimizing equations (15) and (21) together is *O*(d*nl*) in each iteration. Therefore, the overall time complexity of DCH is *O*(*n*^2^+*T*_*c*_*l*+*T*(*n*^3^+d*nl*)). In this work, time complexities *O*(*T*_*c*_*l*) and *O*(d*nl*) can be ignored due to *T*_*c*_,  *l*, *d* ≪ *n* so that our complexity is nearly *O*(*Tn*^3^+*n*^2^). Additionally, the calculation of the hash codes is a linear projection with a time complexity of approximately *O*(1), and the online search can be performed by XOR operations. Although the algorithm proposed in this paper adds a constraint on SMVH, the maximum number of iterations *T* directly affects the time complexity of the algorithm. It can be proven in subsequent experiments that DCH can converge in fewer iterations. Thus, the time complexity of DCH is in a reasonable range.

## 4. Experiments

In this section, we first introduce the datasets used in this paper, and then, the baselines and some experimental details will be introduced. Finally, we present the experimental results.

### 4.1. Datasets

CC_WEB_VIDEO [4] is the most useful dataset in near-duplicate video retrieval (NDVR) research, which contains data from YouTube, Google, and Yahoo. There are 12,877 videos that are divided into 24 sets, and keyframes are extracted by a uniform sampling method to represent the video. Since some videos do not have label information, we take 3,482 videos with labels as the experimental dataset. In each category, we select 70% of the video data as the training set and the remainder as the testing set. We extract 10 keyframes for each video uniformly and extract 4096-dimensional features to represent keyframes by using the pretrained VGG-19 network.

**HMDB51** [38] contains 6,766 human action videos selected from movies and some other public sources such as YouTube. The dataset is divided into 51 categories, and each of them includes approximately 100 clips. In each category, we randomly select 45 video samples. Of these, 25 videos are added to the training set and the rest are select to the testing set. We uniformly extract 10 keyframes for each video, and the VGG-19 pretraining network is used to extract the 4096-dimensional deep features.

**UCF101** [39] contains 13,320 videos which has been divided into 101 human behavior categories, such as sports, instruments, character interactions, and others used for action recognition. We randomly select 70 videos in each category to join the training set, and 30 videos to join the testing set. For each video, 10 keyframes are uniformly selected to represent the video. We use VGG-19 to extract the 4096-dimensional features for each keyframe.

### 4.2. Experimental Setting

#### 4.2.1. Baselines

Several state-of-the-art hash functions, including ITQ [19], SH [20], DSH [21], LFH [22], KSH [23], JMVH [35], and SMVH [34], are used for comparison. Among these methods, ITQ, SH, and DSH are unsupervised hashing methods, while LFH, KSH, JMVH, and SMVH are supervised hashing methods. For the comparative test, we use the source codes published to conduct the experiment. JMVH and SMVH can also be used for multiview video retrieval, but in this paper, we only test these methods as a single view method. It is worth noting that all the experimental results are obtained in MATLAB R2016a on the same computer with an Intel Core i7-6700 CPU @ 3.40 GHz, 72 GB RAM and the 64 bit Windows 10 operating system.

#### 4.2.2. Evaluation Metrics

We use four popular evaluation metrics to comprehensively evaluate experimental results. The mean average precision (mAP) is widely used in the retrieval field. The higher the mAP score is, the better the retrieval performance of the method is. The precision@K curve represents the precision accuracy versus the first *K* retrieved samples, where precision represents the proportion of the number of retrieved correct videos to the total number of retrieved videos. The recall@K curve represents the average recall rate versus the first *K* retrieved samples, where recall represents the proportion of the correct video volume retrieved in all near-duplicate video samples. The precision-recall (PR) curve is an index used to evaluate reliability and is widely used in the fields of medicine and machine learning.

#### 4.2.3. Parameter Selection

We have three model parameters, including *λ*, *μ*, and *γ*, and the number of iterations *T*. According to SMVH [34], we set *λ*=0.9 and *μ*=0.01. As shown in Figure 2(a), when *γ* is in the range of 0.05 to 1, the results are stable across three different datasets. Therefore, we empirically choose *γ*=1 in our proposed model. The maximum number of iterations *T* determines the training time cost and the performance, so it is worth discussing.  Figure 2(b) shows the effect of the maximum iterations *T* in the range of 100 to 1400 on mAP performance. For HMDB51, it can be seen that the best mAP is generated with *T* = 800 before decreasing. However, in the other two datasets, *T*=800 is not an optimal experimental result. Therefore, after comprehensive consideration, *T*=1000 is set as the final parameter setting.

### 4.3. Results and Discussion

Table 1 shows the mAP results for different lengths of hash codes on the three datasets, and the results of other evaluation metrics are shown in Figures 3–5. We will give the detailed analysis of all results of the three datasets in the following parts.

According to Table 1, for the CC_WEB_VIDEO dataset, the mAPs are very high because the dataset is movie clips, and videos of the same category are near-duplicate videos. As shown in Table 1, the performance of the proposed DCH is at least 1.85% better than that of the other methods from 32 to 64 bits. When the code length is 96 bits, the mAP of DCH is slightly lower than that of LFH. As shown in Figure 3, the experimental results of our method in precision@K and recall@K are equal to or slightly higher than those of most other methods. Besides, as the code length increases, the performance of our proposed DCH gradually surpasses that of other methods. Figures 3(i)–3(l) show that the area surrounded by DCH is gradually increasing.

Table 1 shows that our proposed DCH performs better than other hash methods in most cases in the HMDB51 dataset. Although the mAP performance of the JMVH method surpasses 2.39% over that of DCH with 32 bits, the mAPs of our proposed DCH are better than those of the other comparison methods in the subsequent experiments.  Figure 4 shows that when the length of hash codes is larger than 32 bits, regardless of whether precision@K curve, recall@K curve, or PR curve is used, DCH has excellent performance compared with other methods in all metrics for the precision@K curve, recall@K curve, and PR curve.

For the UCF101 dataset, DCH obtained the optimal experimental results in the range of [32, 48, 64] bits. It is worth noting that the size of the UCF101 dataset is relatively large, and SMVH cannot obtain discriminative video hash when the hash code length is very small. Therefore, SMVH has no experimental results available for *l*=32 and *l*=48. As shown in Figure 5, the performance of DCH is much higher than those of some of the methods except JMVH. We can see that the recall rate of DCH for positive samples is slightly lower than that of JMVH based on Figures 5(e)–5(h). Figures 5(i)–5(k) show that the performance of DCH for 32 to 48 bits is better than those of all other methods for the PR curve.

## 5. Conclusion

In this paper, we propose a novel supervised video hashing framework, termed discriminative codebook hashing, which can generate discriminative binary codes for video retrieval. The proposed DCH encourages samples within the same category to converge to the same code word and maximizes the mutual distances between different categories. Specifically, we generate a discriminative codebook to distinguish between samples of different categories more accurately. Extensive experimental results prove that the performance of DCH is significantly improved compared to several state-of-the-art methods. In future work, we will use a smaller matrix storing the similarity information between samples to avoid consuming considerable training time and space when the amount of data is large. This will improve the performance of the model while reducing the time complexity.

## Figures and Tables

**Figure 1:** The framework of DCH. We divide the entire experiment into two steps, namely, offline learning and online retrieval. In the offline phase, we join keyframe features and predefined codebook to learn hash functions. In the online phrase, we map the query video into a set of binary codes through hash functions. Next, we use the exclusive or (XOR) operation to obtain the Hamming distance between the query video and samples in the database. Finally, we take videos with the shortest Hamming distance as the video retrieval results.

**Figure 2:** Parameter analysis on the CC_WEB_VIDEO, HMDB51, and UCF101 datasets. (a) mAP vs. *γ* (weight parameter *γ*) and (b) mAP vs. *T* (iteration parameter *T*).

**Figure 3:** Precision@K (a–d), recall@K (e–h), and PR (i–l) curves on the CC_WEB_VIDEO dataset.

**Figure 4:** Precision@K (a–d), recall@K (e–h), and PR (i)–(l) curves on the HMDB51 dataset.

**Figure 5:** Precision@K (a–d), recall@K (e–h), and PR (i–l) curves on the UCF101 dataset.

**Algorithm 1:** Discriminative codebook.

**Algorithm 2:** Discriminative codebook hashing.

**Table 1:** The mAP of different hash code lengths on three datasets, where the best experimental results are given in bold.

Method	CC_WEB_VIDEO				HMDB51				UCF101			
	32 bits	48 bits	64 bits	96 bits	32 bits	48 bits	64 bits	96 bits	32 bits	48 bits	64 bits	96 bits
ITQ [19]	0.6877	0.7725	0.8099	0.7700	0.0697	0.0749	0.0793	0.0885	0.1383	0.1620	0.1801	0.2119
SH [20]	0.6729	0.7026	0.6994	0.6708	0.0662	0.0657	0.0642	0.0653	0.1033	0.1138	0.1244	0.1395
DSH [21]	0.6510	0.7060	0.6929	0.8158	0.0505	0.0628	0.0671	0.0750	0.0720	0.0667	0.0815	0.1082
LFH [22]	0.8327	0.8088	0.9854	**0.9912**	0.0141	0.0208	0.0148	0.0225	0.0032	0.0038	0.0078	0.0113
KSH [23]	0.9368	0.9030	0.9477	0.8761	0.2470	0.2811	0.3054	0.3144	0.3222	0.3598	0.3972	0.4075
JMVH [35]	0.7842	0.5576	0.4335	0.3745	**0.2807**	0.3015	0.2418	0.1295	0.3941	0.5166	0.6007	**0.6875**
SMVH [34]	0.9346	0.9411	0.9543	0.7490	0.1212	0.1399	0.1374	0.0319	—	—	0.0094	0.0304
DCH	**0.9531**	**0.9763**	**0.9886**	0.9858	0.2568	**0.3819**	**0.3600**	**0.4150**	**0.5310**	**0.6137**	**0.6609**	0.6458

## Data Availability

CC_WEB_VIDEO dataset can be downloaded from http://vireo.cs.cityu.edu.hk/webvideo/, the HMDB51 dataset can be downloaded from https://serre-lab.clps.brown.edu/resource/hmdb-a-large-human-motion-database/#dataset, and the UCF101 dataset can be downloaded from https://www.crcv.ucf.edu/data/UCF101.php.
